# Solitaire™ Stent Thrombectomy System in the Treatment of Acute Lower-Limb Ischemia: Comparisons in Safety and Effectiveness with Conventional Catheter-Directed Thrombolysis Therapy

This article has been retracted.

**DOI:** 10.1155/2022/6997221

**Published:** 2022-09-20

**Authors:** Hao Huang, Jianping Gu, Haobo Su, Liang Chen, Xu He, Jie Kong, Yadong Shi, Zhaoxuan Lu, Yuan Yuan

**Affiliations:** Department of Interventional Radiology, Nanjing First Hospital, Nanjing Medical University, Nanjing, China

## Abstract

**Objective:**

The study aimed to investigate the safety and efficacy of the Solitaire™ AB Stent System (ev3 Inc., Plymouth, MN, USA) for the treatment of acute lower extremity ischemia (ALLI) compared with conventional catheter-directed thrombolytic therapy.

**Methods:**

Retrospective analysis of patients with ALLI treated in the Department of Interventional Radiology at the First Hospital of Nanjing from January 2017 to April 2020 divided into a conventional (CDT) group (*n* = 106) and a percutaneous mechanical thrombectomy (PMT) group (*n* = 55) according to the procedure. PMT was performed using the Solitaire™ AB stent system. The combined clinical outcomes of mortality, major amputation, recurrent ischemia, and major morbidity were compared between the two groups.

**Results:**

Of the 161 patients, 128 (79.5%) did not have a composite clinical outcome after 12 months of follow-up, namely, 78 CDT patients and 50 PMT patients, with significant differences in composite clinical outcome (26.4% vs. 9.1%, *P* = 0.010) and mortality (19.8% vs. 7.3%, *P* = 0.037) between them. Thrombolytic drug dose (19.34 ± 5.93 vs. 13.55 ± 6.54 mg, *P* < 0.001) and length of hospital stay (8.29 ± 3.91 vs. 5.49 ± 1.18 days, *P* = 0.003) were significantly lower in the PMT group.

**Conclusion:**

PMT with the Solitaire™ AB Stent System is safer and more effective in treating patients with Rutherford stage I-IIB ALLI, with the advantage of rapid opening of obstructed vessels, shorter thrombolysis time, reduced thrombolytic dose, and improved blood flow to the infrapopliteal vessels.

## 1. Introduction

Acute lower limb ischemia (ALLI) is a vascular surgical emergency caused by embolism, arterial thrombosis, arterial entrapment, or trauma, resulting in a sudden reduction or interruption of blood supply to the limb, resulting in a drastic reduction of blood supply to the relevant tissues, which can seriously threaten the survival of the limb and even endanger life [1, 2]. Early diagnosis, rapid restoration of lower limb perfusion, and reduction of perioperative mortality and amputation rates are the keys to the treatment of acute lower limb ischemia [3, 4]. The main etiologies of acute lower extremity ischemia include arterial embolism due to embolus dislodgement or arterial thrombosis based on atherosclerosis [5, 6]. With the increasing trend of aging population in China, the incidence of arterial thrombosis on the basis of atherosclerosis has also increased significantly and has gradually surpassed that of arterial embolism [7]. The most common source of embolism in acute arterial embolism is cardiogenic emboli, which account for about 75–80% of emboli, namely, atrial fibrillation, arrhythmia-induced appendage thrombosis after myocardial infarction, redundancy on valves, and intra-atrial mucinous tumors [8]. The typical clinical manifestations are the 6P signs, i.e., limb pain, waxy pallor, decreased skin temperature, pulselessness, abnormal sensation, and paresthesia.

The onset of acute limb ischemia can cause an abrupt interruption of blood supply to the skin, nerves, muscles, and other tissues, as there is not enough time for new blood vessels to grow to compensate for the perfusion of blood to the lower limb [9], which can seriously threaten limb survival. The tolerance of different tissues to ischemic time is different; irreversible damage occurs after 4–6 hours of ischemia in nerves, 6–8 hours in muscle tissues, and 8–12 hours in skin, so we need to develop the appropriate treatment plan quickly according to the degree of ischemia [10].Rutherford's staging [11], one of the clinical staging of ALLI, was proposed in 1986 and updated in 1997. It is based mainly on the assessment of limb appearance, skin temperature, motor and sensory function, and arteriovenous Doppler flow signals to determine whether the limb is alive, threatened, or has developed irreversible damage [12] and classifies ALLI as grades I, IIa, IIb, and III. For patients with Rutherford grade I and IIa ischemia, the appropriate treatment can be selected by performing appropriate tests to determine the cause; for patients with Rutherford grade IIb, immediate hemodynamic reconstruction should be performed, depending on the degree of ischemia, the cause of ischemia, the duration of ischemia, postoperative complications, and the patient's physical condition. Patients with Rutherford grade III may require amputation to save their lives.

The common treatments for acute lower extremity ischemia include surgical and endoluminal treatments, mainly incisional thrombectomy, catheter-directed thrombolysis (CDT), bypass surgery, endarterectomy, percutaneous mechanical thrombectomy (PMT), and hybrid procedures combining two or more surgical modalities [13]. Despite timely thrombolytic therapy or arteriotomy for embolization, amputation occurs in 10% to 15% of patients during hospitalization, and approximately 15% to 20% of patients die within 1 year of onset [14]. There is growing evidence that surgery often fails to achieve satisfactory revascularization due to residual thrombus in the distal vessels and greater surgical trauma, and CDT is thought to be associated with a higher risk of bleeding and a greater incidence of distal embolism, often leading to a poor prognosis [15, 16]. In recent years, the Solitaire™ AB stent for thrombectomy (ev3 Inc., Plymouth, MN, USA) has been widely used in the field of acute ischemic stroke, with recanalization rates of 66%–88% in occluded vessels [17, 18]. A retrospective study showed that mechanical revascularization using the Solitaire™ AB device with manual thrombus aspiration is a fast, safe, and effective way to reduce the requirement for CDT [19]. However, to our knowledge, no studies have compared it with conventional endovascular therapy. Therefore, this study compared the safety and efficacy of Solitaire™ stent thrombectomy with conventional CDT therapy in the treatment of ALLI.

## 2. Materials and Methods

The retrospective clinical study was approved by the ethics committee of Nanjing First Hospital. The medical records of all patients treated at Nanjing First Hospital were archived in the hospital information system database, and patients were selected for enrollment by searching this database from January 2017 to April 2020 according to the inclusion/exclusion criteria of the study. As this was a retrospective study, patient consent was waived.

### 2.1. Inclusion Criteria

Inclusion criteria include (1) patients with a confirmed diagnosis of acute lower extremity ischemia based on clinical presentation, signs, bilateral lower extremity vascular ultrasound, and CTA; (2) onset ≤14 days; (3) no previous history of lower extremity arterial surgery; and (4) complete clinical and imaging data

### 2.2. Exclusion Criteria

Exclusion criteria include (1) contraindications to anticoagulation or thrombolysis, (2) non-acute lower extremity ischemia, (3) treated with vascular bypass surgery, (4) arterial embolism or arterial thrombosis caused by trauma, and (5) no surgical treatment or missing clinical data

Preoperative preparation: For patients suspected of acute lower limb ischemia based on the present medical history and physical examination, relevant investigations should be actively completed after admission, especially the lower limb artery CTA (model: SOMATOM Force) and the ultrasound of both lower limbs to clarify the level of vascular occlusion and the degree of blockage and to assess the ischemia of the lower limbs. If there is no contraindication to anticoagulation, the patient should be given low-molecular heparin anticoagulation therapy immediately. To prevent the development of thrombus from spreading, the patient can be treated with poppy bases to expand blood vessels and improve microcirculation to buy time for blood vessel reconstruction. Anticoagulation should be contraindicated for patients with recent traumatic brain injury, recovery from cerebral hemorrhage, and severe hepatic and renal insufficiency. If the patient has severe pain in the lower limbs, symptomatic treatment such as oxygen, sedation, pain relief, and appropriate rehydration should be given. If the patient is in urgent need of surgical treatment, the surgical mode should be decided according to the patient's ischemic classification, ischemic genesis, systemic condition and imaging data. The patient's surgical risk should be minimized, and the patient and family should be informed of the surgical risks and possible postoperative complications to improve the preoperative preparation.

All procedures were performed under local anesthesia via the ipsilateral femoral artery or contralateral femoral artery approach. After identifying the diseased blood vessels by lower-limb angiography on the lesion side, in the CDT group, a thrombolytic catheter (Medtronic, Inc. Minneapolis, MN, USA) was placed into the thrombotic segment and recombinant tissue plasminogen activator (rt-PA) (Actilyse®; Boehringer Ingelheim, Ingelheim am Rhein, Germany) was subsequently given, followed by infusion with a dose of 0.4–0.85 mg/h through the thrombolytic catheter. Next, lower-limb arteriography was performed every 24 ± 4 h for re-examination. In the PMT group, a Solitaire™ AB stent (6 × 30 mm or 4 × 20 mm) was applied to perform thrombus aspiration of the blood vessels of the diseased segment; then, CDT could be completed after the thrombus load of the diseased segment was relieved (Figure 1). A bolus injection of 5 mg of rt-PA was administered intraoperatively, if necessary.

During thrombolysis, daily detection of hematological indices was conducted, namely, blood cell counts, electrolyte levels, and renal and coagulation functions, and the fibrinogen content was measured at least once a day. The thrombolysis rate was adjusted according to the fibrinogen test results, and the hematological indices were re-examined at the end of thrombolytic therapy. When necessary, endovascular treatment could be used as an auxiliary technique (stent implantation or percutaneous transluminal balloon angioplasty) to restore artificial blood vessels, implants, or blood vessels to be unobstructed and to realize the full perfusion of distal blood vessels. Subcutaneous injection of low-molecular-weight heparin was not performed routinely during thrombolytic therapy, but clopidogrel (75 mg/day) alone or combined with aspirin was given to patients with thromboembolism attributable to arteriosclerosis obliterans for ≥6 months. Warfarin or new anticoagulants were given orally in a continuous manner to patients with atrial fibrillation, cardiac thrombosis, thromboembolism, or unexplained hypercoagulability. In short, personalized decisions were made for different patients, and the aforementioned drugs were used in combination with each other in some patients.

### 2.3. Observation and Follow-Up

After treatment, the patients were followed up with at 1, 6, and 12 months. The primary outcome for analysis was the occurrence of any event of a composite clinical outcome (CCO) during the first year after treatment (1). The occurrence of any of these events was considered an adverse outcome, and the patient was classified as reaching a primary outcome of this study. The components of the CCO included (1) recurrent ischemia; (2) major amputation (above the ankle) or death; (3) life-threatening hemorrhage, either intracranial or blood loss, producing hypotension and requiring resuscitation; and (4) vascular complications, e.g., perforation, occlusion, pseudoaneurysm, or dissection requiring unplanned or emergent surgical repair. The secondary outcomes were the incidence of complications and the runoff score of thrombolytic therapy. The patients were considered to have diabetes mellitus if they were receiving treatment with oral hypoglycemic agents or insulin. Hypertension was defined as a systolic pressure of >140 mmHg or diastolic pressure of >90 mmHg in two or more blood pressure measurements and/or a previous diagnosis of hypertension or the administration of antihypertensive drugs. Hyperlipidemia was defined as any or all elevated blood lipid and/or lipoprotein levels based on hematological examination. Amputation was defined as amputation at or above the ankle. The runoff score (0–19) was determined according to the Society for Vascular Surgery guidelines, with higher scores indicating greater obstruction of the popliteal and inferior genital arteries [20].

### 2.4. Statistical Analysis

The SPSS statistical software package (version 18.0; IBM Corporation, Armonk, NY, USA) was adopted for statistical analysis. Normally distributed data are expressed as mean ± standard deviation values, while qualitative data are expressed as frequencies (percentages). Furthermore, the *t* test was used to compare the measured data between two groups, and Fisher's exact test or the chi-squared test was used to compare numerical data between the groups. Then, we visualized analysis results using the R software (version 3.0.2; R Foundation for Statistical Computing, Vienna, Austria), and subgroup analysis was performed according to the Kaplan-Meier method.

## 3. Results

From January 2017 to April 2020, a total of 161 patients were enrolled in this study. Of these, 106 patients were treated with CDT (CDT group) and 55 patients with ALLI who underwent Solitaire™ stent thrombectomy (PMT group) were obtained to compare the treatment effectiveness with CDT. The mean age of the patients was 72.51 years (standard deviation, 8.76 years; range, 49–93 years), and the study included 84 men (52.2%) and 77 women (47.8%). The classification scheme of acute limb ischemia was as follows: 9 cases of Rutherford I, 89 cases of Rutherford IIa, and 63 cases of Rutherford IIb. There was no significant difference in baseline data between the 2 groups except in the number of patients with hyperlipidemia. The baseline data are presented in Table 1.

The treatments performed in the CDT and PMT groups are summarized in Table 2. At the 1-year follow-up, the event rate for the CCO in the CDT group was 26.4% compared to that of 9.1% in the PMT group (*P* = 0.010). In terms of the CCO, the groups showed significantly different rates of death (19.8% vs. 7.3%; *P* = 0.037) and life-threatening hemorrhage (15.1% vs. 3.6%; *P* = 0.029). Between the two groups, there was no significant difference in major amputation (3.8% vs. 1.8%; *P* = 0.498), ongoing/recurrent ischemia (1.9% vs. 1.8%; *P* = 0.976), or vascular complications (1.9% vs. 1.8%; *P* = 0.976). Two fasciotomies were performed following the completion of thrombolytic therapy in the CDT group. Moreover, five more patients in the CDT group and one patient in the PMT group developed an intracranial or gastrointestinal hemorrhage and died within days of their procedure. The percentage of patients who underwent stenting significantly differed between the CDT and PMT groups (45.3% vs. 27.3%, *P* = 0.026), and significant differences were found in thrombolytic duration (38.09 ± 14.20 vs. 24.56 ± 10.98 h, *P* < 0.001) and rt-PA thrombolytic dose (19.34 ± 5.93 vs. 13.55 ± 6.54 mg, *P* < 0.001) between the groups. Technical success was achieved for 91 patients in the CDT group and 54 patients in the PMT group (85.9% vs. 98.2%, *P* = 0.013).

Regarding fibrinogen levels, there was no significant difference between the CDT and PMT groups before treatment (2.99 ± 0.50 vs. 2.98 ± 0.57 g/L, *P* = 0.221), but an obvious difference was observed after treatment (1.54 ± 0.63 vs. 1.82 ± 0.53 g/L, *P* = 0.041). Considering hemoglobin content, we failed to find a significant difference between the CDT and PMT groups before (104.77 ± 11.19 vs. 108.05 ± 11.25 g/L, *P* = 0.609) or after (90.90 ± 13.46 vs. 95.85 ± 12.19 g/L, *P* = 0.594) treatment. The runoff score did not differ between the CDT and PMT groups before treatment (13.28 ± 2.32 vs. 13.44 ± 2.57 points, *P* = 0.384), whereas it was significantly higher in the CDT group after treatment (7.19 ± 3.25 vs. 5.53 ± 1.84 points, *P* < 0.001).

At 1-year follow-up, Kaplan-Meier estimates of the proportion of CCO were greater in the CDT group than in the PMT group (*P* = 0.015; Figure 2(a)). In the subgroup analysis, Kaplan-Meier estimates of the proportion of patients without AF disease or CCO did not differ significantly between treatment groups (89.5% in the CDT group and 93.3% in the PMT group; *P* = 0.664; Figure 2(b)). In contrast, in the atrial fibrillation subgroup, Kaplan-Meier estimates of the CCO-free rate at 12 months were higher in patients treated with CDT than in those treated with PMT (70.1% in the CDT group versus 90.0% in the PMT group; *P* = 0.023; Figure 2(c)). In patients with Rutherford classification I–IIa, there was no significant difference in CCO rates between the two groups (Figure 2(d)), but significantly more patients with Rutherford classification IIb had CCO in the CDT group compared with the PMT group (Figure 2(e)).

## 4. Discussion

Acute lower extremity ischemia is a common clinical vascular surgical emergency that can seriously affect the life of the patient and the survival of the affected limb if the patient is not treated with timely intervention. It is one of the most common causes of amputation, with approximately 1.5 amputations in 10,000 people per year [21]. Amputation rates in patients with acute lower extremity ischemia have been documented to range from 10% to 15% and 30-day mortality rates from 15% to 25% [22]. The outcome of the affected limb in patients with acute lower limb ischemia is related to the duration of lower limb ischemia, and the longer the duration of ischemia, the higher the risk of the affected limb facing necrosis. Therefore, timely hemodialysis is important for such patients. The duration of lower extremity ischemia in patients with lower extremity atherosclerosis and atherothrombosis varies from a few hours to several months. Since atherosclerosis is a progressive process, the affected extremity has developed a rich collateral circulation during the long-term ischemia and is able to tolerate a longer period of ischemia. The diversity of clinical presentations combined with the complexity of the arterial wall structure makes it difficult for clinicians to evaluate and treat these patients.

The current clinical treatment of acute lower extremity ischemia is divided into three main categories: (1) surgical thrombectomy (ST) with Fogarty catheter; (2) catheter-directed thrombolysis (CDT); (3) noninvasive and minimally invasive percutaneous mechanical thrombectomy (PMT). Percutaneous mechanical thrombectomy (PMT) and hybrid treatment (HT) combine intracavitary therapy with surgical thrombectomy and multiple methods of thrombectomy. Both incisional thrombectomy and catheter-contact thrombolysis are important treatment modalities for patients with acute lower limb ischemia. Incisional thrombectomy with balloon catheter-based thrombectomy maximizes the removal of femoropopliteal artery thrombus in patients with acute lower extremity ischemia but has little effect on the embolization of some small arteries below the knee. Repeated embolization is more likely to damage the intima of the artery and cause secondary thrombosis after surgery, which aggravates the ischemia of the affected limb. Catheter-contact thrombolysis technique has a high success rate, is well tolerated by patients, and is equally effective for some small branches of the infrapopliteal artery and thrombus in the microcirculation and is increasingly used in acute lower limb ischemic diseases [23]. Due to the high risk of recent bleeding and distal embolism with catheter contact thrombolysis, it is often used clinically in combination with other techniques to reduce the risk of bleeding.

The Solitaire™ AB stent is a widely used technology in the field of cerebral ischemic stroke and has been shown to be effective in patients who do not respond well to thrombolytic therapy. Interestingly, a large body of evidence suggests that the Solitaire™ AB stent can rapidly remove dislodged emboli, open the vessel, and improve the efficiency of thrombolysis and that the Solitaire™ AB stent is suitable for a wide range of vessel sizes with a minimum available vessel diameter of 1.5 mm, suggesting that it can be applied to emboli in distal branches of lower extremity arteries [24, 25]. Rapid opening of the vessel is important in patients with ALLI, but thrombolysis is often less effective in some patients (e.g., those with atrial fibrillation) due to the stiff texture of the emboli. The Solitaire™ AB stent allows for rapid removal of the emboli, thereby opening the outflow tract and improving the efficiency of thrombolysis. This may explain why the Solitaire™ AB stent works better in AF and in the Rutherford IIb subgroup.

This study found that Solitaire™ AB stenting can significantly improve the prognosis of ALLI patients while reducing the thrombolysis time and the runoff score. The device displays the advantages of quickly opening blocked vessels, restoring blood flow, and improving the efficiency of thrombolysis. This study's results illustrated that compared to the CDT group, the CCO rate, mortality, thrombolysis time, thrombolytic agent dose, and length of hospital stay were significantly reduced in the PMT group; meanwhile, PMT had obvious advantages concerning postoperative fibrinogen levels and the runoff score. It is well known that lower runoff scores indicate improved blood flow in below-the-knee vessels, and a large number of studies have also confirmed that increased blood flow in below-the-knee vessels improves the long-term effect of lower-extremity arterial therapy [26, 27].

This study has some drawbacks. (1) This study has certain limitations, being a single-center, retrospective study, not a randomized controlled study, and there may be information bias and selection bias in the collection of study subjects, which may have an impact on the study results. (2) In general, the cases collected in this study were of high age, with many comorbid diseases, and mainly patients with Rutherford ischemic classification of grade II, which may not accurately reflect the actual situation and overall prognosis of the disease, and a large sample and multicenter study is still needed to obtain relatively accurate results. (3) The operators in this study were not the same person, and since each person has different surgical methods and techniques, this may have an impact on surgical decision making, surgical outcomes, postoperative complications, and reintervention rates. It is hoped that homogeneity will be ensured in future studies to minimize errors.

## 5. Conclusion

Acute lower extremity ischemia is a common disease in vascular surgery and often threatens the life safety of the patients and the survival of the limb. It requires the receiving physician to make the correct diagnosis and choose the correct treatment in the shortest possible time. In summary, PMT with Solitaire™ AB stent is safe and effective in treating patients with Rutherford stage I-IIB ALLI. This strategy is characterized by rapid opening of blocked vessels, shortened thrombolysis time, reduced thrombolytic dose, and improved blood flow to the infrapopliteal vessels.

## Figures and Tables

**Figure 1:** Bracket legend. Note: (a) Angiography shows acute below-the-knee artery occlusion, (b) Solitaire™ AB stent insertion through the below-the-knee arteries, (c) angiography after mechanical thrombo-aspiration revealed patency, and (d) macroscopic aspect of the aspirated thrombi.

**Figure 2:** Kaplan-Meier cumulative event curves at 12 months of follow-up. Note: (a) overall cohort, (b) no atrial fibrillation subgroup, (c) atrial fibrillation disease subgroup, (d) Rutherford classification I–IIa subgroup, and (e) Rutherford classification IIb subgroup.

**Table 1:** Patient baseline data.

Parameters	CDT group (*n* = 106)	PMT group (*n* = 55)	*P* value
Age (years)	72.99 ± 9.06	71.56 ± 8.09	0.328
Gender (%)	—	—	0.817
Male	56 (52.8%)	28 (50.9%)	—
Female	50 (47.2%)	27 (49.1%)	—
Affected limb (%)	—	—	0.664
Left	54 (50.9%)	30 (54.5%)	—
Right	52 (49.1%)	25 (45.5%)	—
BMI (kg/m^2^)	22.19 ± 2.93	22.74 ± 2.54	0.238
Symptom duration (h)	45.38 ± 24.94	39.93 ± 28.47	0.212
Rutherford classification	—	—	0.289
I	8 (7.6%)	1 (1.8%)	—
IIa	56 (52.8%)	33 (60.0%)	—
IIb	42 (39.6%)	21 (38.2%)	—
History of smoking	42 (39.6%)	23(41.8%)	0.788
History of past illness	—	—	—
Atrial fibrillation	87 (82.1%)	40 (72.73%)	0.168
Rheumatic heart disease	1 (0.9%)	2 (3.6%)	0.269
Hypertension	74 (69.8%)	34 (61.8%)	0.306
Diabetes mellitus	33 (31.1%)	19 (34.6%)	0.660
Renal dysfunction	21 (19.8%)	12 (21.8%)	0.765
Cerebral infarction	19 (17.9%)	13 (23.6%)	0.389
Malignant tumor	17 (16.0%)	8 (14.6%)	0.804
Hyperlipidemia	81 (76.4%)	33 (66.0%)	0.030∗
Proximal embolism site	—	—	0.365
Iliac artery segment	3 (2.8%)	4 (7.3%)	—
Femoral artery segment	26 (24.5%)	15 (27.3%)	—
Popliteal artery segment/popliteal–distal artery	77 (72.6%)	36 (65.5%)	—

Notes: CDT: catheter-directed thrombolysis; PMT: percutaneous mechanical thrombectomy; BMI: body mass index.

**Table 2:** Treatments, complications, and treatment outcomes of patients in the CDT and PMT groups.

	CDT group	PMT group	*P* value
Stenting	48 (45.3%)	15 (27.3%)	0.026∗
Thrombolysis duration (hours)	38.09 ± 14.20	24.56 ± 10.98	<0.001∗
rt-PA dosage (mg)	19.34 ± 5.93	13.55 ± 6.54	<0.001∗
Technical success	91 (85.9%)	54 (98.2%)	0.013∗
Length of hospital stay(days)	8.29 ± 3.91	5.49 ± 1.18	0.003∗
Composite clinical outcome	28 (26.4%)	5 (9.1%)	0.010∗
Death	21 (19.8%)	4 (7.3%)	0.037∗
Major amputation	4 (3.8%)	1 (1.8%)	0.498
Recurrent ischemia	2 (1.9%)	1 (1.8%)	0.976
Life-threatening hemorrhage	16 (15.1%)	2 (3.6%)	0.029∗
Vascular complication	2 (1.9%)	1 (1.8%)	0.976

Notes: CDT: catheter-directed thrombolysis; PMT: percutaneous mechanical thrombectomy; rt-PA: recombinant tissue plasminogen activator.

## Data Availability

The original contributions presented in the study are included in the article. Further inquiries can be directed to the corresponding author.
